The article "A Review on the Use of Microsoft Kinect for Gait Abnormality and Postural Disorder Assessment" was published in 2021. Journal: J Healthc Eng.

# A Review on the Use of Microsoft Kinect for Gait Abnormality and Postural Disorder Assessment

**DOI:** 10.1155/2021/4360122

**Published:** 2021-11-01

**Authors:** Anthony Bawa, Konstantinos Banitsas, Maysam Abbod

**Affiliations:** Department of Electronic and Electrical Engineering, College of Engineering, Design and Physical Sciences, Brunel University, UB8 3PH, Uxbridge, UK

## Abstract

Gait and posture studies have gained much prominence among researchers and have attracted the interest of clinicians. The ability to detect gait abnormality and posture disorder plays a crucial role in the diagnosis and treatment of some diseases. Microsoft Kinect is presented as a noninvasive sensor essential for medical diagnostic and therapeutic purposes. There are currently no relevant studies that attempt to summarise the existing literature on gait and posture abnormalities using Kinect technology. The purpose of this study is to critically evaluate the existing research on gait and posture abnormalities using the Kinect sensor as the main diagnostic tool. Our studies search identified 458 for gait abnormality, 283 for posture disorder of which 26 studies were included for gait abnormality, and 13 for posture. The results indicate that Kinect sensor is a useful tool for the assessment of kinematic features. In conclusion, Microsoft Kinect sensor is presented as a useful tool for gait abnormality, postural disorder analysis, and physiotherapy. It can also help track the progress of patients who are undergoing rehabilitation.

## 1. Introduction

Microsoft's Kinect sensor is a motion-sensing device that gives users the features to interact with game consoles and computers via ways such as gestures, spoken commands, or movement [1]. Kinect sensors provide new and enhanced features for motion detection and 3D reconstruction. Kinect sensors also introduce many features that allow for more accurate research into the movement of the human body and its gestures. The sensors allow for interaction through voice commands that is a unique component of the technology. It has detectors and infrared emitters to capture human physical activities.

The key components of Microsoft Kinect sensors are the RGB cameras, IR depth sensors, and the multiple microphone array. The second version of Kinect has some enhanced features compared to earlier Kinect [2]. The colour camera of Kinect v2 has 1,920 × 1,080 @30fps while that of Kinect v1 has 640 × 480 @30fps. In terms of the depth camera capabilities, Kinect v2 uses 512 × 424 pixels, while Kinect v1 uses 320 × 240 pixels, and as a result, Kinect v2 has better image recognition compared to the earlier version. Kinect v2 is noted to have a wider area view compared to Kinect v1. Another key feature is that Kinect v2 has better skeletal joint tracking where it is able to capture 26 joints, whereas Kinect v1 can only capture 20 joints. The unique feature of Kinect sensors can be applied to the medical field for the purposes of diagnosing diseases and physiotherapy rehabilitation of people who may have walking disabilities due to physical injury or related diseases.

As stated above, Kinect has found application in many areas related to posture and motion capturing. The major bulk of studies are related to Kinect research in the areas of motion tracking, monitoring, diagnosis, and rehabilitation. Some representative studies with Kinect technology include: Lavanya et al. [3] presented dynamic finger gestures with skeletal data extracted from the depth sensor. A unique technique was designed for the recognition of dynamic gestures that can be used in auditoriums and classrooms. This approach allowed for more dynamic hand gestures to be developed that can be used in different environments. An example is a tutor using this technique to instruct students in a classroom who have speech problems to assist in their studies.

The use of Kinect for medical monitoring and diagnosis has also been trialed by researchers. Ales Prochazka et al. [4] presented a novel technique of using Kinect for heart rate estimation and breath monitoring to determine the likelihood of any medical condition. The mean thorax movement was monitored within a selected area to estimate the breathing of patients. Huy-Hieu et al. [5] presented a real-time system for the detection of objects for patients who are visually impaired. A unique system was designed that allowed visually impaired people to move freely and to detect any obstructions. Object detection was based on the 3D information captured with a depth sensor. However, the designed system was limited to only indoor use. Xin Dang et al. [6] presented a novel interactive system with an electroencephalogram and depth sensor for people with dementia. Skeletal data captured from the depth sensor were extracted to determine the motion of a user and their mental state. The designed system using a deep neural network can be used to aid patients with dementia. Torres et al. [7] provided a novel approach to assist physicians in the diagnosis of Parkinson's disease using posture and movement captured with Kinect. The characteristics of movements such as frequency and amplitude were essential to study tremors in people with Parkinson's. The results achieved in the study can assist clinicians to diagnose Parkinson's based on the tremors intensity and the postural changes.

Kinect sensors are also widely used for the purposes of rehabilitation. Capecci et al. [8] demonstrated an innovative approach in the evaluation of dynamic movement in a rehabilitation scenario. They were able to track skeletal joints in evaluating the performance of patients during a low back pain physiotherapy exercise. Postolache et al. [9] developed a unique framework for physiotherapy assessment based on a mobile application using skeletal data. The designed system assists physiotherapists to improve the effectiveness of the training sessions for patients undergoing rehabilitation. Monique Wochatz et al. [10] illustrated a reliable and valid assessment of the lower extremity rehabilitation of exercises using Kinect v2 sensors. The authors demonstrated the Kinect sensor as a reliable tool in assessing the lower limb position and the joint angles during exercises. Sanjay et al. [11] developed a unique framework for stroke rehabilitation of patients in a home environment. A framework was designed to aid patients who have suffered a stroke in their treatment process. The designed system can be used indoors to help patients who have difficulty in movement.

Abnormal gait is the asymmetric movement of a person that is most likely to be caused by disease or physical injuries. This could be a result of nerves damage, injuries, weakness of muscles, or joint problems. The detection of gait abnormalities at an early stage can help prevent other complications. There are traditional wearable sensors for gait abnormal detection; however, these conventional methods are quite cumbersome to use. Kinect is seen as a better alternative to wearable sensors in gait abnormal detection.

As such, gait analysis has also received wide interest among researchers [12–14]. Kinematic features such as the step length, walking speed, and cadence are useful to determine the gait of an individual. This will normally be cyclical and symmetric unless there are some forms of abnormalities. The human gait could be affected by the musculosketal and neurological systems as well as the motions habits [15]. Hassain Bari et al. [16] presented a novel method by designing a deep neural network for gait recognition. This was then evaluated with a 3D skeletal gait data set. Another study by Wan Zharfan et al. [17] illustrated an economic technique of gait analysis based on pixel coordinates of body joints. The technique served as an alternative method to determine gait parameters in a Vicon motion analysis.

The human posture is the physical positioning by which the body takes at a particular time. Posture is the arrangement of the structure of the human body and its position. Correct body posture can help reduce pressure on the human body by keeping it balanced. The human body posture may be intentional or unintentional due to natural causes. There are several techniques for postures recognition with skeletal data. Samiul Monir et al. [18] presented a novel technique with a rotation and scale-invariant for posture recognition from skeletal features. This technique for posture recognition used skeletal data and angle rotation of an individual. A set of vectors and manipulation of angles were used to determine the posture. Zequn et al. [19] developed a novel posture recognition model that can be used to identify different postures captured. The depth sensor was used to generate features of different body parts of an individual. The captured features were then fed into the support vector machine (SVM) to identify the posture.

Although there are quite a number of studies available using Kinect for the assessment of gait and posture abnormalities, to the best of our knowledge, there is no overall review study that attempts to summarise articles on the use of the Kinect sensor for gait abnormality and posture disorder assessment. Our review adopts a systematic approach similarly used by Shmuel Springer et al. [20]. The study provides up-to-date review of the articles for analysis and discussion.

## 2. Methods

In this section, we retrieve articles that meet the inclusion criteria for our study. The existing articles identified were summarised into tables indicating the methods used and the sampling area. The sample area stated the source from which the article was retrieved, the authors of the article, and the year it was published. Our focus was on articles that used Kinect sensors for assessing gait and posture abnormalities.

### 2.1. Search and Identification of Articles

The scholarly database used to identify the articles were: IEEE Xplore, ScienceDirect, CINAHL plus, and PubMed. The search was done in two different parts as follows:

- Part 1: the use of Kinect sensors for the detection of gait abnormality or disorder
- Part 2: the use of Kinect sensors for detection posture disorder or instability

The key terms used in part 1 of the search were: “Kinect sensor,” “gait abnormality,” “gait disorder,” and “walking abnormality.” In the second part, the key terms used were: “Kinect sensor,” “posture disorder,” “posture abnormality,” and “posture instability.” The search was conducted between January and May 2021 to retrieve the most recent articles.

### 2.2. Eligibility Criteria of the Identified Articles

In identifying the articles for the study, we conducted two different searches for the database by two independent authors. The authors were able to identify and remove duplicate articles from the various database. The elimination of irrelevant articles was done without bias or oversight in order to get all relevant articles that meet the inclusion criteria. A number of diseases that could affect gait and posture abnormalities were included. They were: Parkinson's, ataxia, multiple scoliosis, stroke, and depression.

The exclusion criteria were for articles that only discussed gait detection and postures without considering abnormality. In the second part, articles that only discuss posture assessments without examining posture disorder or deformity were also not included. Articles that used wearable sensors for gait abnormality and posture disorder detection were not included.  Figure 1 is a flowchart diagram of the search methodology.

## 3. Results

The initial search and retrieval of all articles from the various database were 458 for gait and 283 for posture, all using Kinect technology. The articles were further screened to ensure they meet the eligibility criteria for this study. In the end, a total of 26 articles were included for gait abnormality and 13 articles for posture disorders.

Table 1 summarises all the studies that were included for the review for gait abnormality, the journals where the articles were retrieved and the year of publications. In Table 1, the methodology describes the sampling method applied, the statistical method, and the descriptive approach used. That sampling method describes the number of participants in the study, gender, and age distribution. The disease associated with the abnormality was stated. The sampling methods from the reviewed articles were categorised as fully stated, partially, or not stated. The statistical method describes the statistical techniques that were used in the analysis of the data. The statistical methods were either sufficiently used or partially used. It describes the models and mathematical equations that were used in the analysis of skeletal data. The description method used refers to capturing of the skeletal data, processing of data, algorithms used, and the analysis of the results. It also includes the tools used in the analysis of results and a detailed discussion of the findings. Finally, the description method was either adequate or partial description.

The approach used in Table 1 was also similarly adopted in Table 2 except that it summarised the various articles for identifying posture disorders using Kinect. The sampling methods, statistical methods, and the description method are also indicated in this table.

In Table 3, the details of each article included in the study were categorised into two major phases. The first phase deals with the sampling technique used in each study while the second phase describes the key gait features captured with the major findings of each study. The limitations for each study were also included in the table.

A total number of 26 articles were reviewed. Most of the articles stated the number of participants in the study except in [26,28,37,42,43,45]. The majority of the studies used Kinect v2 as the main tool for capturing skeletal data for gait abnormality assessment, while a few articles used the older Kinect v1. In [37,44], the Asus Xtion PRO was used as a gold standard with a Kinect sensor for capturing skeletal data. Most of the reviewed articles did not state the data analysis tool. However, in [22,25,29,31,35,39,40], MATLAB was explicitly stated as the main tool for data analysis. In [23], the SPSS package was used as the data analysis tool. The gait features captured were mainly the step/stride length (m), stride time (s), gait speed (m/s), gait cycle (deg), gait rhythm (m/s), and step time (s). Some of the key joint angles measured were the hip, knee, and the ankle. Various algorithms were used to train the models for gait abnormality detection.

A total number of 13 articles were included for the assessment of posture abnormality or disorder. Some of the reviewed articles [42,46,50,51] did not state the participants in the studies. In Table 4, Kinect v2 was mostly used for skeletal data capturing, except in a few studies that used Kinect v1. Nine of the reviewed articles used Kinect v2 while four used Kinect v1. Most of the studies did not state any medical condition that resulted in posture abnormality. However, in [47], Parkinson's disease was stated, and in [56], a case of chronic traumatic brain injury was present. In [50,58], patients with suspected multiple scoliosis were also assessed for posture abnormality. The majority of the reviewed articles did not state the data analysis tool except in [47,48,50] that stated MATLAB. In [58], the IBM Watson Analytics was used to analyse the data for posture abnormality for patients with suspected cases of multiple scoliosis.

## 4. Discussion

### 4.1. Gait Abnormality or Disorder

The purpose of this study is to review the available studies using Microsoft Kinect for the assessment of gait and posture abnormalities. The key features measured included the angles formed by leg swing, speed, and distance of each gait step. These parameters were useful in detecting gait asymmetry in order to distinguish normal from abnormal gait. Some other components from the summarised studies were the algorithms used, the major findings of each study, and limitations.

From the reviewed articles, various methods were employed in assessing and detecting gait abnormality. The gait features captured were mainly the step/stride length (m), gait speed (m/s), gait cycle (deg), and step time (s). Some other gait features captured from the studies were angles of knee joints, ankle joints, and hip angles joints. The measured joint angles were used to train the models in detecting gait abnormalities. The measurement of joint angles helped improve the efficiency and robustness of the trained models to detect gait abnormality.

They were various algorithms used to train the models for gaits abnormality detection. Some of the algorithms used in Table 3 were machine learning algorithms. The machine learning algorithms were either supervised or unsupervised, depending on the approach used. Supervised machine learning algorithms use classifications and regressions, while unsupervised use clustering and associations to determine outliers in the data. Algorithms that were used in the designed models for gait abnormality were: Bayesian algorithm, K-nearest neighbors algorithm (KNN), convolutional neural network (CNN), recurrent neural network (RNN), long short-term memory (RNN-LSTM), isolated forest (IF) algorithm, and one-class support vector machine (OC-SVM) algorithm. Depending on the algorithm that was used and the mythological approach, different accuracy were achieved. The Bayesian algorithm was commonly used in [15, 19, 23, 33] for the assessment of gait abnormalities. RNN-LSTN algorithm was used in three of the studies [20, 36, 37, 40]. Amr Elkholy et al. used unsupervised one-class support vector machine (OC-SVM) and isolated forest algorithms for abnormal detection in [31, 33]. Some other algorithms such as the EDSS and MSWS were also applied in [27]. The algorithms used in the various studies cannot be compared to determine which is more efficient and robust. This is because different methods and data sets were used to achieve the desired accuracy.

The general limitation of the summarised studies has to do with the relatively small data set used. Most of the studies did not use a large data set to test the robustness of the trained model except in [21, 22, 25, 29, 33, 34, 44] that used large data sets. Another limitation was some gait parameters were not used in training the models for abnormal gait assessment. Some studies did not also include key joint angles in the trained model. Therefore, some of the models did not give high precision and robustness in assessing gait abnormalities. Also, the use of Kinect v1 has limited capabilities compared to Kinect v2 that has more enhanced 3D skeletal tracking capabilities.

### 4.2. Posture Abnormality or Disorder

From Table 4, some body features were measured to determine the posture abnormality of a person. They were the body center mass position and the shoulder position angulation. The head position and the neck angles were also essential to detect postural instability. In [47,49], the center of body mass was used to determine the postural instability. The rapid upper limb assessment (RULA) method was commonly used to assess postural instability in [52,57]. The distance between the neck, shoulder blade, and angles was very essential in determining the abnormal posture of a person. In [52], the height, hips, and shoulder position were measured as well as the shoulder angles. In [53], the knee joints, ankle joints, the lateral joints, and interior joints were computed. The spine angle was also used in [47] to determine the abnormal posture of an individual.

Different algorithms were used to determine postural disorder from the summarised studies. The algorithms that were used included pattern recognition neural algorithm, CoVNet model, Berg balance scale (BBS) method, and the RULA technique. These algorithms were used to track the static body position features and key joint angles to determine the postural instability of a person. The accuracy in the detection of posture disorder was not considered because the studies focused only on determining if there was posture abnormality.

The limitations of the various summarised studies largely depended on the small data set used in the various studies.

### 4.3. Mathematical Analysis of Gait Abnormality

In Sun Bie et al. [21], the spatial position was used with the associated joints for each subject walking. The extracted joint angle formed were then calculated. The equations used in the joint angle computation were given by the following equation:

(1) $$\begin{array}{c} \text{len}\left(i,k\right)=\left\|J\left[i\right]-J\left[k\right]\right\|,\\ \theta \left(i,k,j\right)=\cos^{-1}\frac{\left(J\left[i\right]-J\left[k\right]\right)*\left(J\left[j\right]-J\left[k\right]\right)}{\left\|J\left[i\right]-J\left[k\right]-J\left[j\right]-J\left[k\right]\right\|}, \end{array}$$

where *J[i]* represents the joints, *len (i*,*k)* represents the distance between joint *i*, and *kθ(i*, *k*, *j)* describes the angle formed by joint *i*, *k*, and *j*. Therefore, the angles formed by the left leg and the right leg were calculated by the following equation:

(2) $$\begin{array}{c} R_{s}=\rho \left(\theta_{l},\theta_{r}\right)\\ =\frac{Ε\left[\left(\theta_{l}-m_{\theta l}\right)*\left(\theta_{r}-m_{\theta r}\right)\right]}{\sqrt{Ε\left(\theta_{l}-m_{\theta l}\right)*Ε\left(\theta_{r}-m_{\theta r}\right)}}, \end{array}$$

where *θ*_*l*_ and *θ*_*r*_ represents the angles formed on the left and right leg, respectively, of a subject walking and E(∗)represents the expected value of the operation for the simulation. The equations were used in computing the key joint angles to determine gait asymmetry. The angles calculated were the hip angle, knee angle, and the ankle angle. The challenge with this technique is that there may be some difficulties in measuring the inner joint angles of subjects. The gait cycles were computed and given by the following equation:

(3) $$\begin{array}{c} T_{s}=\frac{1}{n-1}\sum_{i=2}^{i=n}\left|x_{i}-x_{i}-1\right|*0.0333, \end{array}$$

where |*∗*| is the absolute value from the operation and 0.0333 is the conversion factor from the Kinect sensor.

In [37], the gait energy image (GEI) was used based on the Gaussian mixture model (GMM) for each pixel in the simulation. The GEI was the image captured with the Kinect sensor of an individual in a walkway. It can be used to determine the dynamic information of a gait sequence. The gait cycle was then extracted and computed at the point where a normalised autocorrelation from the silhouette image was high in the GEI.

(4) $$\begin{array}{c} C\left(N\right)=\frac{\sum_{x,y}\sum_{n=0}^{k}S\left(x,y,n\right)S\left(x,y,n+N\right)}{\sqrt{\sum_{x,y}\sum_{n=0}^{k}S{\left(x,y,n\right)}^{2}\sqrt{\sum_{x,y}\sum_{n=0}^{k}{\left(x,y,n+N\right)}^{2}}}}, \end{array}$$

where *C(N)* represents the autocorrelation for *N* frameshift, and the *N* value is chosen to empirically represent all the abnormal gait cycles that exist in the tested data sets; *K = N*_*Total*_*–N–1* where *N*_*Total*_ represents the total number of frames sequence. *S(x*, *y*, *n)* indicates the pixel values at a position *(x*,*y)* in the silhouette frame *n*. The GEI was then computed as an average of the normalised and aligned silhouette over the gait cycle in the following equation:

(5) $$\begin{array}{c} G\left(x,y\right)=\frac{1}{n_{\text{cycle}}}\sum_{i=1}^{n_{\text{cycle}}}S_{i}\left(x,y\right), \end{array}$$

where *n*_cycle_ represents the frame of the gait cycle while *S*_*i*_ is the silhouette frame of *x*, y pixel coordinates of the image captured. The extracted gait energy image (GEI) and the gait cycle were used to determine gait abnormality from different viewing points based on the colour image sequence. However, this technique does not consider factors that may affect the colour image sequence such as clothes variations.

In [32], the Euclidian distance was used to compute the joints and dynamic body parts for a subject to determine gait abnormality. The Euclidian distance is defined in the following equation, where the distance *r* and *s* are the shortest distance between the line segment *rs*:

(6) $$\begin{array}{c} d\left(r,s\right)=d\left(s,r\right)\\ =\sqrt{{\left(r_{x}-s_{x}\right)}^{2}+{\left(r_{y}-s_{y}\right)}^{2}+{\left(r_{z}-s_{z}\right)}^{2}}. \end{array}$$

Hero's formula was then used to calculate the triangular area of the gait cycle. The area obtained by Hero's formula is given by the following equation:

(7) $$\begin{array}{c} \text{Area\_of\_triangle}=\sqrt{{\left(r_{x}-s_{x}\right)}^{2}+{\left(r_{y}-s_{y}\right)}^{2}+{\left(r_{z}-s_{z}\right)}^{2}}. \end{array}$$

The step length was then calculated between the right foot from left foot in the Euclidian distance as follows:

(8) $$\begin{array}{c} \text{step\_length}=\sum_{i=1}^{n}\sqrt{A+B}, \end{array}$$

where *A* and *B* are defined as the area formed by the joint angles.

The areas and angles were formed between the hip right foot and the left foot. A triangle was generated to get the area and angle between the right foot. Therefore, the Euclidean distance to compute for the maximum foot distance lifted from the ground is given by the following equation:

(9) $$\begin{array}{c} {\text{Ground}}_{\text{clearance}}=\max\left(\text{right}\_{\text{foot}}_{y}\right)-\min\left(\text{right}\_{\text{foot}}_{y}\right). \end{array}$$

The limitations in using the Euclidean distance for computation has to do with the multiple dimensions and the sparse nature of data. This presents some variations in trying to measure the gait distances for subjects in a walkway.

In [44], asymmetry features were used to detect walking abnormality in a subject. The motion asymmetry between the right body parts and the left body parts of the skeletal data was extracted. The average distance extracted from the skeletal data for a pair of joint angles was then computed. The Euclidean distance used to represent the asymmetry feature was calculated from the following equation:

(10) $$\begin{array}{c} D_{ij}^{p}=\frac{\sum_{t=1}^{n}\sqrt{{\left(x_{it}-x_{jt}\right)}^{2}+{\left(y_{it}-y_{jt}\right)}^{2}+{\left(z_{it}-z_{it}\right)}^{2}}}{n}, \end{array}$$

where *D*^*ρ*^ represents the left and right of the average distance of a subject while x_it_, y_it_, and z_*it*_ represents the 3D coordinates of the joint *i* of a subject of frame *t* and *n* is the number of frames of action sequence. *N*_p_ is the set of joints for the left and right body parts of an individual. The velocity magnitude feature was computed in the study to detect slow action performed by the subject. The equation used to calculate is as follows:

(11) $$\begin{array}{c} V=\frac{\sum_{t=1}^{n-1}\sum_{i=1}^{N}\sqrt{{\left(x_{i\left(t+1\right)}-x_{it}\right)}^{2}+{\left(y_{i\left(t+1\right)}-yit\right)}^{2}+{\left(z_{i\left(t+1\right)}-z_{it}\right)}^{2}}}{\left(n-1\right)N}. \end{array}$$

Equation (11) is essential in computing the displacement magnitude for each body joint between two successive frames where *N* represents the number of joints and *n* represents the number of frames.

In [27], gait assessment of a patient was evaluated by extracting the time series for the knee angles and the gait cycle of dynamic time warping (DTW). The knee DTW distance and the hip were then calculated and averaged to get the mean DTW distance of individual patients. The mean DTW distance for the hip joints and the knee that are denoted by D_*HP*_ and D_*KP*_ are defined by the following equations:

(12) $$\begin{array}{c} D_{KP}≔\frac{1}{2}\left[\frac{1}{m_{p}n_{c}m_{c}}\overset{m_{p}}{\underset{j=1}{\sum }}\overset{n_{c}}{\underset{q=1}{\sum }}\sum_{r=1}^{m_{c}}\text{DTW}\left(\theta_{LK_{i,t}},\phi_{LK_{q,r}}\right)+\frac{1}{m_{p}n_{c}m_{c}}\sum_{j=1}^{m_{p}}\sum_{q=1}^{n_{c}}\sum_{r=1}^{m_{c}}\text{DTW}\left(\theta_{RK_{i,t}},\phi_{RK_{q,r}}\right)\right], \end{array}$$

(13) $$\begin{array}{c} D_{HP}≔\frac{1}{2}\left[\frac{1}{m_{p}n_{c}m_{c}}\sum_{j=1}^{m_{p}}\sum_{q=1}^{n_{c}}\sum_{r=1}^{m_{c}}\text{DTW}\left(\theta_{LH_{i,t}},\phi_{LH_{q,r}}\right)+\frac{1}{m_{p}n_{c}m_{c}}\sum_{j=1}^{m_{p}}\sum_{q=1}^{n_{c}}\sum_{r=1}^{m_{c}}\text{DTW}\left(\theta_{RH_{i,t}},\phi_{RH_{q,r}}\right)\right]. \end{array}$$

### 4.4. Equations for Postural Abnormality Assessment

Several researchers have proposed different techniques for the recognition of the human posture and 3D human reconstruction. The posture probability density is used to reconstruct the posture of human beings [60]. It is based on human body measurement that can be used to determine posture. This is used as a density estimator in the following equation:

(14) $$\begin{array}{c} \hat{p}\left(x;h,\gamma \right)=\sum_{n=1}^{N}\gamma_{n}\kappa \left(\frac{x-x_{n}}{h}\right), \end{array}$$

where *K(*.) is the kernel, *h* is the bandwidth of the kernel, and *d* is the degree of freedom of the data. The probability density estimate is then given by the function where the weights *γ* in each kernel are based on the reduced set density estimation (RSDE).

The RULA-based method is a common technique for posture assessment of an individual. This technique can be used to determine the postural abnormality of an individual. Two techniques are used to calculate the joint angles, which are input from a module score. These techniques use a voxel-based angle estimation in which the RULA score for the upper joints is computed based on their location. The joint angles are computed using vectors that are dependable on the location of each joint with correspondence to the parent joint location. This is given by the angle between two vectors of the parents' joints and the child's joints in the following equation:

(15) $$\begin{array}{c} \theta =\;\cos^{-1}\frac{p_{1}.p_{2}}{\left\|p_{1}\right\|.\left\|p_{2}\right\|}. \end{array}$$

The magnitude of the two vectors *P*_*1*_ and *P*_*2*_ are calculated by:

$\left\|p_{1}\right\|=\sqrt{p_{1}.p_{1}}$ and $\left\|p_{2}\right\|=\sqrt{p_{2}.p_{2}}$, where the computed value is then submitted into equation (15). The RULA method is a good technique for posture assessment because it is easy and fast to use. This can be used in the evaluation of posture disorder without the need to conduct any experimental measurements. This technique is, therefore, significant to conduct risks of musculoskeletal disease with regard to the posture of an individual.

## 5. Conclusion

In this study, we presented Microsoft Kinect as a noncontact tool for the assessment of gait abnormality and posture disorder. While there are several studies on gait recognition, only a few have dealt with the assessment of gait and posture abnormalities. Early detection of gaits and posture abnormalities plays a significant role for clinicians to provide corrective rehabilitation measures. Even though this is a comprehensive study, there may be some articles that are not included.

In our study, we presented 26 studies for gait abnormality assessment and 13 articles for posture disorder. The summarised studies differ by the methodology used, the gait features extracted, and the analytical tools used to process the skeletal data. Different algorithms were applied in the summarised studies, and some of them made use of machine learning algorithms. The results showed what has been done so far in the area of gait and posture abnormality assessment.

From our analysis, Kinect sensors have a high success rate of approximately 87% in abnormalities assessment. It has an accuracy ranging between 83% and 98.1% from the summarised articles for gait abnormality. This is quite acceptable in the clinical settings for the purposes of diagnosis of diseases associated with gait and posture disorders. Although Microsoft has stopped the release of Kinect sensors, it is still an important tool for diagnostic purposes. It can be concluded that Kinect sensor is an essential monitoring tool for use in medical diagnostics and can also help track the progress of patients who are undergoing rehabilitation.

## Figures and Tables

**Figure 1:** Flowchart for the search methodology of articles included.

**Table 1:** Reviewed articles on gait abnormality or disorder.

Sample study area			Methodology used for the reviewed articles		
Authors	Journal/conference paper	Year of publication	Sampling method in study	Statistical method	Description method
Bei et al. [21]	IEEE sensors journal	2018	Partially stated	Sufficiently used	Adequate description
Wang et al. [22]	IEEE sensors journal	2019	Fully stated	Sufficiently used	Adequate description
Tsukagoshi et al. [23]	Journal of clinical neuroscience	2019	Fully stated	Sufficiently used	Partial description
Amin amini et al. [24]	Journal of healthcare engineering	2019	Fully stated	Sufficiently used	Adequate description
Prochazka et al. [25]	Elsevier – digital signal processing	2015	Partially stated	Partially used	Partial description
Pachón-Suescún et al. [26]	International journal of electrical and computer engineering (IJECE)	2020	Partially stated	Partially used	Partial description
Gholami et al. [27]	IEEE journal of biomedical and health informatics	2016	Fully stated	Partially used	Adequate description
Maxime devanne et al. [28]	International conference on pattern recognition (ICPR)	2016	Not stated	Not used	Adequate description
Latorre et al. [29]	Elsevier – journal of biomechanics	2018	Fully stated	Partially used	Adequate description
Prakash et al. [30]	IEEE transactions on instrumentation and measurements	2021	Fully stated	Partially used	Adequate description
Nguyen et al. [31]	Sensors, MDPI	2016	Partially stated	Sufficiently used	Adequate description
Shrivastava et al. [32]	Elsevier – materials today: Proceedings	2020	Partially stated	Partially used	Partial description
Prochazka et al. [33]	IEEE international conference on image processing (ICIP)	2014	Partially stated	Partially used	Partial description
Fang et al. [34]	IEEE access on multiphysics	2019	Fully stated	Sufficiently used	Adequate description
Ismail et al. [35]	IEEE international conference on advances in biomedical engineering (ICABME)	2017	Partially stated	Not used	Partial description
Amini et al. [36]	Disability and rehabilitation: Assistive technology	2018	Fully stated	Sufficiently used	Adequate description
Elkholy et al. [37]	IEEE journal of biomedical and health informatics	2019	Not stated	Partially used	Partial description
Soltaninejad et al. [38]	Sensors, MDPI	2019	Fully stated	Partially used	Adequate description
Kozlow et al. [39]	Sensors, MDPI	2018	Fully stated	Sufficiently used	Adequate description
Chakraborty et al. [40]	International conference on computational science	2020	Partially stated	Partially used	Partial description
Jyothsna et al. [41]	IEEE engineering in medicine and biology society (EMBC)	2020	Partially stated	Not used	Partial description
Won et al. [42]	IEEE engineering in medicine and biology society (EMBC)	2019	Not stated	Not used	Partial description
Jinnovart et al. [43]	IEEE conference on decision and control (CDC)	2020	Not stated	Not used	Partial description
Elkholy et al. [44]	International conference of the IEEE engineering in medicine and biology society (EMBC)	2020	Fully stated	Not used	Adequate description
Meng et al. [45]	Joint conference on computer vision, imaging and computer graphics theory and applications	2016	Not stated	Not used	Partial description
Jun et al. [46]	IEEE access	2020	Not stated	Not used	Partial description

**Table 2:** Reviewed articles on posture abnormality or disorder.

Sample study area		Methodology used for the reviewed articles			
Authors	Journal/Conference	Year of publication	Sampling method in study	Statistical methods	Description of model used
Ferrais et al. [47]	Sensors, MDPI	2019	Fully stated	Sufficiently used	Adequate description
Jawed et al. [48]	IEEE international conference on emerging trends in engineering, sciences and technology	2019	Not stated	Not used	Partial description
Yang et al. [49]	IEEE sensors	2014	Fully stated	Sufficiently used	Partial description
Castroa et al. [50]	Elsevier porto biomedical journal	2016	Fully stated	Partially used	Adequate description
Chin-hsuan et al. [51]	Sensors, MDPI	2020	Fully stated	Sufficiently used	Adequate description
Abobakr et al. [52]	IEEE international conference on systems, man, and cybernetics	2017	Partially stated	Not used	Partial description
Napoli et al. [53]	Biomedical engineering society	2017	Partially stated	Partially used	Partial description
Meng-Che shih et al. [54]	Journal of neuro engineering and rehabilitation	2016	Fully stated	Sufficiently used	Adequate description
Chanpimol et al. [55]	Archives of physiotherapy	2017	Partially stated	Partially used	Partial description
Bortone et al. [56]	IEEE-EMBS international conference on biomedical and health informatics	2014	Not stated	Not used	Partial description
Modesto et al. [57]	Elsevier applied ergonomics	2017	Partially stated	Not stated	Partial description
Norbert et al. [58]	Health informatics meets eHealth	2017	Fully stated	Fully stated	Adequate description
Rose et al. [59]	Elsevier: gait and posture	2012	Partially stated	Not stated	Partial description

**Table 3:** Detailed features of articles on gait abnormality or disorder.

Sampling techniques				Key gait features and aims of the identified articles						
Authors	Gender and age range of participants	Abnormality or disease	Kinect sensor version	Data type capture	Gait parameters measured	Data analysis tool	Algorithm used	Accuracy achieved (%)	Major findings	Limitations of study
Bei et al. [21]	Gender and age not stated	70 normal walking and 50 walking disorder	Kinect v2	Skeletal data	Leg swing angle (deg), knee and ankle joint angle (deg), step length (m), gait cycle (deg)	Not stated	K-means algorithms, Bayesian algorithms	Not stated	A novel technique was designed to demonstrate movement disorder through gait symmetry analysis	Some key gait parameters and joint angle were not considered. Only a small data set was used to test the model
Wang et al. [22]	98 individuals; gender and age not stated	Depression	Kinect v2	Skeletal data	Gait velocity (m/s), *Joint angles (deg)*	MATLAB	t-SNE algorithm	93.75	A nonintrusive framework was designed to detect depression	Some gait features are required to improve the robustness of the model in a real environment
Tsukagoshi et al. [23]	Ataxia (male = 14 female = 11); age 54.1 ± 14.6 years. Parkinson's (male = 10 female = 15); age 68.4 ± 8.1 years. Healthy people (male = 13 female = 12), age 62.0 ± 13.9 years	25 Patients with ataxia, 25 patients with Parkinson's, and 25 health people	Kinect v2	Skeletal data	Stride length (m), feet length (m), gait rhythm, (m/s)	SPSS package suit	Clinical scale	Not stated	Kinect depth sensor to quantitatively evaluate gait interference for patients who have a movement disorder	Body joint gaits angulation were not considered and thus there may be less precision with this model
Amini et al. [24]	15 participants (12 male and 3 female); average age 54–92 years	People with Parkinson's	Kinect v2	Skeletal data	Gait cycle (deg), knee angle (deg), number of footsteps (m)	Not stated	Heuristic fall detection algorithm	Not stated	A unique model was designed to detect freeze of gait for people with Parkinson's	The developed system is limited to only the *x*-axis for the freeze of gait detection
Aleš prochazka et al. [25]	51 individuals; gender not stated; age: Parkinson's, 52–87 years, healthy mature: 32–81 years, young: 23–25 years	18 Individuals with Parkinson's, 18 healthy matured, and 15young ones	Kinect v1	Not stated	Step length (m), gait length (m/s), stride length (m)	MATLAB	Bayesian algorithm	94.1	A novel technique was developed using Bayesian classification algorithm to recognise gaits disorder for people with Parkinson's disease	Some key joint angles were excluded in developing an abnormal gait recognition model and thus not so efficient
Cesar et al. [26]	Gender and age not stated	Not stated	Kinect v2	Skeletal data	Step speed (m/s), stride speed	MATLAB	LSTM algorithm	98.1	A model was designed to detect gait abnormality using the LSTM algorithm	Body joint angles are required to test and improve the accuracy of the model
Gholami et al. [27]	MS (male = 1, female = 9); age = 41–79 years. NP (male = 1, female = 9); age 36–80 years	10 multiple scoliosis and 10 normal people	Kinect v2	Skeletal data	Gait velocity (m/s), stride length (m), stride time (s), step time (s)	Not stated	EDSS algorithm and MSWS algorithm	Not stated	A novel framework was designed to evaluate the gaits abnormality of people with multiple scoliosis	The designed framework does not provide enough reliability to detect the disease. There is less accuracy with the designed model.
Devanne et al. [28]	Gender and age not stated	Not stated	Kinect v2	Skeletal data	Step length (m), body joint angles (deg)	Not stated	Riemannian manifold algorithm	Not stated	A model is designed to detect gait abnormality using motion trajectories	The method is not able to identify static gait abnormality such as a freeze of gait
Latorre et al. [29]	45 healthy individuals (men = 31, women = 14); age 30.6 ± 7.6 years. 38 stroke survived people (men = 22, women = 16); age = 56.1 ± 13.2 years	45 Healthy individuals and 38 stroke surviving people	Kinect v2	Skeletal data	Gait speed (m/s), stride length (m), stride time (s), swing time (s), step time (s), step asymmetry	MATLAB	Bayesian algorithm	Not stated	The authors illustrated the reliability of using Kinect-based methods to estimate gait disorder for poststroke adult individuals	The method used in the study were limited which influenced some errors with the gait parameters measured
Prakash et al. [30]	24 individuals (13 males and 11 females); age not stated	Not stated	Kinect v2	Skeletal data	Left knee angle (deg), right knee angle (deg)	Not stated	IR-UMB algorithm	Not stated	A model was developed to detect gait abnormality using contactless IR-UWB	Only the knee angle was considered and this may not give accuracy of the designed model
Nguyen et al. [31]	20 individuals; gender and age not stated	10 healthy people and 10 abnormal (Parkinson's/stroke)	Kinect v2	Skeletal data	Left hip angle (deg), right hip angle (deg), left knee angle (deg), right knee (deg), left ankle (deg), right ankle (deg)	MATLAB	HMM algorithm	90.12	A novel approach was designed for gait abnormality detection using skeletal-based data with no prior knowledge of individual gait	The method used in the study provided enough precision of the results achieved
Shrivastava et al. [32]	24 individuals; gender and age not stated	12 Normal walking and 12 abnormal walking	Kinect v1	Skeletal data	Step length (m), gait cycle (s), hip left foot angle (deg), right foot angle (deg)	MATLAB	KNN algorithm, SVM algorithm, and decision tree algorithm	83.33	The authors developed a model using machine learning for gaits abnormality detection using data from Kinect	The model used does not provide high precision and efficiency for detecting gait abnormality
Prochazka et. Al [33]	36 individuals; gender not stated; people with Parkinson's: age = 52–87 years, healthy control: age = 32–81 years	18 Individuals with Parkinson's. 18 healthy control	Kinect v1	Skeletal data	Stride length (m),	MATLAB	Skeletal tracking algorithm	90	A system was designed to detect Parkinson's disease based on the gaits features. This could be used for early detection of Parkinson's.	Only a few parameters such as stride length were used and this does not provide enough efficiency and reliability of the model
Fang et al. [34]	3,669 individuals (1555 males and 2114 females); age range 22–28 years	Suspected cases of depression	Kinect v2	Skeletal data	Walking speed (m/s), arm swing (mm), stride length (m), vertical head position (deg)	MATLAB	SVM algorithm; KNN, RF, and LR algorithms; linear discriminant analysis (LDA)	91.58	A novel model was designed using different ML to detect depression prevalence among students	Different viewing points were not considered in developing a model to detect depression
Ismail et al. [35]	11 individuals; gender not stated; age = 21–25 years	11 healthy control individuals	Kinect v2	Skeletal data	Gait speed (m/s), stride length (m), right knee angle (deg), left knee angle (deg), right ankle (deg), left ankle (deg), hip angle (deg)	MATLAB	Angle average algorithm	Not stated	A novel system is developed to determine gait abnormalities using gait cycle	There were some marginal errors in the data set used that does not provide enough efficiency of the model used in detecting abnormality
Amin amini et al. [36]	11 healthy subjects; age range 24–31 years	Not stated	Kinect v2	Skeletal data	Body angle (deg), feet/joint distance	Not stated	Pythagorean theorem	Not stated	A unique model is designed for casting automatic/dynamic visuals for people with Parkinson's disease	The designed model is limited to indoor environment use
Elkholy et al. [37]	Gender and age not stated	Not stated	Kinect v2, Asus Xtion PRO	Skeletal data	Gait speed (m/s), gait cycle (deg), stride length (m)	Not stated	OC-SVM algorithm and IF algorithm	Not stated	A new approach was designed to detect gait abnormality based on unsupervised gait energy image (GEI)	Some factors that could affect the accuracy of abnormal gaits detection based on the GEI were not considered
Saltaninejad et al. [38]	5 individuals (4 males and 1 female); average age = 30.8 years	Not stated	Kinect v2	Skeletal data	Gait speed (m/s), hip angle (deg), knee angle (deg)	Not stated	Best removal algorithm for FOG	90	An automatic and fast assessment for FOG was designed	The model needs to be tested with real P.D patients to improve its reliability
Kozlow et al. [39]	21 Males and 9 females; age = 25 ± 5.2 years	28 Healthy individuals	Kinect v2	Skeletal data	Cadence (step/min), left angle joint angle (deg), left knee joint angle (deg), right angle joint angle (deg), right knee joint angle (deg), left stride (deg), right stride length (deg)	MATLAB	Bayesian algorithm	88.68	The authors demonstrated the use of Bayesian network algorithm to classify gait abnormality	There are some limitations to the robustness and accuracy of this framework in detecting gait abnormality
Chakraborty et al. [40]	15 individuals; gender and age not stated	Patients with cerebral palsy	Kinect v2	Skeletal data	Gait cycle (deg), left ankle (deg), right ankle (deg)	MATLAB	Dempster shafer classifier	87.5	A novel technique is designed based on automated gait to detect gait abnormality for patients with cerebral palsy	This technique could be challenging in a real environment
Jyothsna et al. [41]	20 individuals; gender not stated; age = 80 years and above	20 people making up the various group, cognitive healthy individuals (CHI), subject cognitive impaired (SCI), and possible mildly cognitive person (pMCI)	Kinect v2	Skeletal data	Stride length (m), mean stride (m), step time (min), cadence (m), gait velocity (m/s)	Not stated	Convolutional neural network algorithm	Note stated	A framework was designed to detect the gait abnormality for patients with dementia	More gaits parameters need to be extracted to test the model on a large data set for dementia patients to improve the efficiency
Deok-won et al. [42]	Gender and age not stated	Not stated	Kinect v2	Skeletal data	Stride length (m), lower limbs body joint angles (deg)	Not stated	RNN-LSTM algorithm	97	The abnormal gait recognition model was designed that is capable of recognising five different abnormal gaits patterns using multiple Kinect sensors	The challenge with this model is that it can only recognise abnormal gait that were used in the training of the RNN-LSTM model. Some abnormal gaits may not be recognised.
Jinnovart et al. [43]	Gender and age not stated	Not stated	Kinect v2	Skeletal data	Stride length (m), body joint angles	Not stated	RNN algorithm, LSTM algorithm, and GRU algorithm	RNN = 73.4, LSTM = 82.8, and GRU = 81.6	A real-time recognition of abnormal gait was presented using recurrent neural network	Some abnormal gait may not be recognised with the designed model
Amr et al. [44]	43 individuals; gender for abnormal gait: male = 19 and female = 13; age = 18–85 years. Healthy control people (male = 8 and female = 3); age = 27–64 years	32 Patients with gait abnormality and 11 healthy control people	Kinect v2, Asus Xtion PRO	Skeletal data	Gait cycle (deg), swing phase(deg), step length (deg)	Not stated	OC-SVM algorithm and IF algorithm	Not stated	A robust and efficient skeletal system was developed to detect abnormal activities performed by a person	The model will require a large data set to test the efficiency of the designed model
Menget al. [45]	Gender and age not stated	Not stated	Kinect v2	Skeletal data	Interskeletal joint distance	Not stated	Random forest classifier	Not stated	A system was developed using a skeletal inter-joint distance to detect abnormal gait and normal gait	The developed system may not be robust because only a few gait features were used on small data sets for abnormal gait detection
Jun et al. [46]	9 individuals; gender and age not stated	1 normal person and 8 abnormal gait	Kinect v2	Skeletal data	Left hip angle (deg), right hip angle (deg), left knee angle (deg), right knee (deg), left ankle (deg), right ankle (deg)	Not stated	RNN algorithm and LSTM algorithm	Not stated	An extraction method feature was developed using RNN to increase the performance of gait abnormality from a skeletal base system	A small data set was used to test the model, and this does not provide high efficiency for gait abnormal detection

RNN: recurrent neural network; LSTM: long short-term memory; GRU: gated recurrent units; OC-SVM: one-class support vector machine; IF: isolation forest; HMM: hidden Markov model; and KNN: k-nearest neighbors.

**Table 4:** Detailed features of articles on posture abnormality or disorder.

Sampling techniques				Key body features and aims of the identified articles					
Authors	Gender and age of participants	Abnormality/disease	Kinect sensor version	Data type capture	Body features measured	Data analysis tool	Algorithm used	Major findings	Limitations of the study
Ferrais et al. [47]	14 individuals (8 male and 6 female); age = 53–80 years	Parkinson's disease	Kinect v2	Skeletal data	Centre of body mass (m)	MATLAB	KNN algorithm	A system is designed for the automatic posture analysis of people with Parkinson's to determine postural instability	More subjects are required to test the model to improve its reliability and efficiency
Jawed et al. [48]	Gender and age not stated	Not stated	Kinect v1	Skeletal data	Body joint angles (deg), body position (m)	MATLAB	Pattern recognition neural algorithm	A system was developed using pattern recognition neural network model that is capable of analysing the whole body of a patient to determine if there is any postural disorder	Not much efficiency with this model in detecting postural disorder with high accuracy
Yang et al. [49]	18 individuals, 9 males and 9 females; age = 24.0 ± 0.7 years	Not stated	Kinect v2	Skeletal data	Centre of body mass (m)	Not stated	RSM algorithm	A system was designed to evaluate the standing balance to determine posture instability	There may be some variations in the calibration to measure the COM
Castroa et al. [50]	98 individuals (males = 50 and females = 48) average; age 24.7 years	Suspected scoliosis disease	Kinect v2	Skeletal data	Shoulder angulations (deg)	MATLAB	SA method	The Kinect sensor was used to quantitatively evaluate the posture of the spine to determine if there is any posture instability	The challenge was that the S2's spinal exposition process was unassured
Chin-Hsuan Liu et al. [51]	45 individuals (15 youth and 30 elderly); age of youth = 24.06 ± 2.02 years; age of elderly = 71.13 ± 4.56 years	Not stated	Kinect v2	Skeletal data	Body joint angles (deg), center of body mass (m)	Not stated	Mediolateral (ML) algorithm	A system was designed to investigate the postural instability using the body joint coordination patterns	Only the mediolateral (ML) motion direction is considered in determining impairments of an individual
Abobakr et al. [52]	Gender and age not stated	Not stated	Kinect v2	Skeletal data	Body joint angles (deg)	Not stated	ConVnet algorithm, AlexNet CNN algorithm, and RULA method	A system was developed using Kinect and for the early detection of postural work-related disorders for people in a manufacturing industry	The methods used only considered the joint angles in designing the model and thus the may not be enough precision
Alessandro Napoli et al. [53]	15 individuals (7 male and 8 female); age not stated	Not stated	Kinect v2	Skeletal data	3D position of body distance (m), spine angle (deg)	Not stated	Balance detection algorithm	A system was designed to determine balancing deficits and postural instability of individuals	There should be an expansion of the features of automatic assessment of postural stability in determining the postural instability
Meng-Che shih. Et l. [54]	Gender BBE (male = 9 and female = 1); gender BT (male = 7 and female = 3); age BBE group 67.5 ± 9.96 years; age BT group 68.8 ± 9.67	Individuals with Parkinson's disease balance-based exergaming group (*N* = 10), balance training group (*N* = 10)	Kinect v2	Skeletal data	Limit of stability (LOS), one leg stance (OLS)	Not stated	BBS method	The authors used a novel technique to assess the postural stability of individuals with Parkinson's disease	The sample size was small, and calibration variability was observed in the exergaming session
Chanpimol et al. [55]	1 individual (1 male); age = 37 years	Chronic traumatic brain injury (TBI)	Kinect v2	Skeletal data	Body position distance (m)	Not stated	Limits of stability (LOS) algorithm	A study to improve the dynamic balance of an individual with TBI and improve the postural instability.	The designed system is limited to a single individual with TBI
Bortone et al. [56]	Gender and age not stated	Not stated	Kinect v1	Skeletal data	Joint angles (deg)	Not stated	Nonasymmetric pattern	An innovative system was designed to identify postural abnormalities using a two-stage approach	The body features measured do provide enough reliability and precision in detecting postural abnormality
Modesto et al. [57]	Gender and age not stated	Not stated	Kinect v2	Skeletal data	Body position (m), joint angles (deg), motion sequence (deg)	Not stated	RULA method	A system was developed using Kinect v2 to detect awkward postures in real time	This designed model needs further investigation to determine its behaviour in a real working environment
Norbert et al. [58]	30 individuals (male = 18 and Female = 12); average age = 16 years	30 students suspected of scoliosis	Kinect v1	Skeletal data	Height measurement of hips and shoulders, angle of hips and shoulder (deg)	IBM Watson analytics	Nonirradiate body tracking method	The detection of scoliosis from students due to their incorrect posture	The confusion matrix used showed Kinect sensor may not provide accurate screening of data captured
Rose A. et al. [59]	20 individuals; gender and age not stated	20 healthy subjects	Kinect v1	Skeletal data	Body joint angles, knee joint, ankle joint, lateral/anterior joint angles	Not stated	Regression algorithm	A postural control assessment to determine those with postural control and those with postural imbalance	Measuring the internal and external joints rotations had limitations, and thus, there are some variations of the results

BBS: Berg balance scale; CNN: convolutional neural networks; RULA = rapid upper limb assessment; and SA: shoulder angulation.

## Data Availability

The data that support the findings of this review paper can be sourced from the summarised table in the study and the references provided.
